# SLC26A4 Mutation Promotes Cell Apoptosis by Inducing Pendrin Transfer, Reducing Cl^−^ Transport, and Inhibiting PI3K/Akt/mTOR Pathway

**DOI:** 10.1155/2022/6496799

**Published:** 2022-08-29

**Authors:** Xiang Dai, Jun Li, XiJiang Hu, Jian Ye, WenQian Cai

**Affiliations:** ^1^Eugenic Genetics Laboratory, Wuhan Children's Hospital (Wuhan Maternal and Child Healthcare Hospital), Tongji Medical College, Huazhong University of Science and Technology, Wuhan 430016, China; ^2^Department of Otolaryngology, Wuhan Children's Hospital (Wuhan Maternal and Child Healthcare Hospital), Tongji Medical College, Huazhong University of Science and Technology, Wuhan 430016, China

## Abstract

**Objective:**

Pendrin is encoded by SLC26A4, which is expressed in the apical membrane of inner ear epithelial cells and drives chloride reabsorption in the apical septum. In the inner ear, pendrin dysfunction and hypofunctional mutations lead to vestibular aqueduct (EVA) enlargement and sensory neural hearing loss. Mutations in SLC26A4 are a common reason of deafness. However, the underlying mechanisms of SLC26A4 mutants in hearing loss remain unknown.

**Methods:**

In the present study, pEGFP-N1 carrying wild-type and mutant SLC26A4 (c.85G>A, c.2006A>T, and c.853G>A) were transfected into HEK-293T cells. GFP fluorescence and GFP levels were determined. SLC26A4 mRNA levels were examined by quantitative real-time polymerase chain reaction (qRT-PCR). Then, the expression of chloride intracellular channel 1 (CLIC1) and CLIC2 was measured by Immunofluorescence assay. Intracellular chloride concentration and apoptotic rate were analyzed by flow cytometry. The levels of membrane/cytoplasmic pendrin, apoptosis-associated proteins, and the PI3K/Akt/mTOR pathway members were determined by Western blot.

**Results:**

Constructed SLC26A4 mutant 1 (c.85G>A), SLC26A4 mutant 2 (c.2006A>T), and SLC26A4 mutant 3 (c.853G>A). The wild-type and 3 mutations were stably expressed in HEK-293T. SLC26A4 mRNA expression was significantly increased after transfection with wild-type SLC26A4 and mutant SLC26A4 compared with the untransfected vector group (*P* < 0.01). Compared with the vector group, the expression levels of membrane pendrin, cytoplasmic pendrin, CLIC1, CLIC2, Bcl-2, p-PI3K, p-Akt, and p-mTOR were upregulated. Compared with the vector group, the chloride concentration, cell apoptotic rate, and the expression levels of caspase-3, caspase-9, and Bax were downregulated. Compared with the vector group, the above effects of SLC26A4 were reversed after the SLC26A4 mutant.

**Conclusion:**

After SLC26A4 mutation, pendrin was transferred from the membrane, the chloride intracellular channel function was reduced, and the excessive accumulation of chloride in the cytoplasm induced cell apoptosis by inhibited PI3K/Akt/mTOR pathway phosphorylation.

## 1. Introduction

Hearing loss is a serious public health issue, affecting nearly 360 million people worldwide according to the report of World Health Organization (WHO) in 2012 [1]. Hearing loss can affect people of all ages. Many risk factors are associated with hearing loss, including genetic mutations, age, noise exposure, ototoxic medication exposure, and infections [2]. More than 120 genes participate in hearing loss, including SLC26A4 gene [3]. SLC26A4 gene, also known as *PDS* gene, encodes a multifunctional anion exchanger pendrin, a protein with 780 amino acids [4]. Pendrin is expressed in several tissues, including the thyroid and kidney, as well as epithelial cells of the inner ear [5, 6]. Mutations in SLC26A4 are the second most frequent cause of hereditary hearing loss in human, after *GJB2* gene mutations [7]. It has been reported that mutations in SLC26A4 are responsible for both Pendred syndrome and non-syndromic hearing loss with enlarged vestibular aqueduct [8]. To date, more than 539 mutations in SLC26A4 gene have been identified [9]. However, the possible molecular mechanism of SLC26A4 mutation in hearing loss has not yet been fully elucidated.

The phosphatidylinositol 3-kinase (PI3K)/Akt/mammalian target of the rapamycin (mTOR) signaling pathway is activated in human cancers, which participates in many cellular processes, such as cell survival, metastasis, autophagy, metabolism, and angiogenesis [10]. Despite the correlation with human cancers, the PI3K/Akt/mTOR pathway is also responsible for the pathogenesis of many other human diseases, such as osteoarthritis, stroke, asthma, and traumatic brain injury [11–14]. Recently, Li et al. have reported that activation of the Akt/mTOR signaling pathway is associated with cochlear hair cell regeneration from supporting cells [15]. However, it is still not clear whether mutations in SLC26A4 lead to hearing loss via regulation of the PI3K/Akt/mTOR pathway.

In the present study, three recombinant plasmids with different SLC26A4 mutants (c.85G>A, c.2006A>T, and c.853G>A) were generated to investigate the underlying mechanism of SLC26A4 mutations in hearing loss.

## 2. Materials and Methods

### 2.1. Mutant Construction

Mutations in SLC26A4 (c.85G>A, c.2006A>T, and c.853G>A) were conducted using Fast Site-Directed Mutagenesis Kit (TIANGEN, Beijing, China) according to the manufacturer's instructions and confirmed by DNA sequencing (TIANYI HUIYUAN Co., Ltd., Wuhan, China). Then, wild-type (coding region of SLC26A4 cDNA) (NM_000441) and mutant SLC26A4 were inserted into eukaryotic expression vector pEGFP-N1 to generate recombinant plasmids containing wild-type, mutant 1 (c.85G>A), mutant 2 (c.2006A>T), and mutant 3 (c.853G>A).

### 2.2. Cell Culture

Human embryonic kidney 293T (HEK-293T) cells were kindly supplied by Shanghai Cell Bank, Chinese Academy of Sciences (China). They were maintained in Dulbecco's Modified Eagle Medium (DMEM) (HyClone, Waltham, MA, USA) with 10% fetal bovine serum (FBS) (Gibco, Grand Island, NY, USA) at 37°C in 5% CO_2_.

### 2.3. Transient Transfection

The cells seeded onto 6-well were cultured at 37°C until growing to 70% confluence. Afterwards, 4 *μ*g pEGFP-N1 vector containing wild-type or mutant SLC26A4 (c.85G>A, c.2006A>T, and c.853G>A) was transfected into HEK-293T cells using Lipofectamine 2000 (Invitrogen, Carlsbad, CA, USA) according to the manufacturer's instructions. Four hours later, culture supernatant was discarded and the cells were further cultured up to 48 h. Green fluorescence of GFP was observed with an inverted fluorescence microscope (Leica, Wetzlar, Germany) and images were taken with this microscope.

### 2.4. Quantitative Real-Time Polymerase Chain Reaction (qRT-PCR)

Total RNA was extracted from HEK-293T cells using TRIzol reagent (Ambion, Austin, TX, USA) according to the manufacturer's instructions. Reaction of cDNA synthesis was conducted using Moloney Murine Leukemia Virus (MMLV) Reverse Transcriptase (TaKaRa, Tokyo, Japan) and ligo (dT)_18_ primer was used in this reaction. Afterwards, qRT-PCR reaction was performed on CFX Connect System (Bio-Rad, Hercules, CA, USA) with SYBR Green PCR Kit (KAPA Biosystems, Boston, MA, USA). Primers used in this study were synthesized by TIANYI HUIYUAN Co., Ltd (Wuhan, China) and these primers were listed below: SLC26A4, 5′-GTTATCTGGGTGTTTACG-3′ (Forward) and 5′-GTGCTAGGGATGCTTC-3′ (Reverse); GAPDH, 5′-CCACTCCTCCACCTTTG-3′ (Forward) and 5′-CACCACCCTGTTGCTGT-3′ (Reverse). The relative expression of SLC26A4 was calculated using 2^−*ΔΔ*Ct^ method.

### 2.5. Western Blot

The membrane and cytosolic proteins were extracted from homogenized cells using Membrane and Cytosolic Protein Extraction Kit (Beyotime, Haimen, China) according to the manufacturer's instructions. Total proteins were extracted from HEK-293T cells lysed by RIPA buffer (Solarbio, Beijing, China). Protein concentration was determined using BCA Protein Assay Kit (Solarbio). Afterwards, 12% SDS-PAGE was prepared to separate the membrane, cytoplasmic, or total proteins (loading protein samples: 20 *μ*g). The proteins in the gel were then transferred to PVDF membranes (Millipore, Bedford, MA, USA). The membranes were incubated with 5% non-fat milk in phosphate-buffered saline (PBS) with 0.05% Tween 20 (PBST) at 4°C overnight. Primary antibody against GFP (1 : 1000; Bioswamp, #MAB43850, Wuhan, China), pendrin (1 : 2000; Bioswamp, #PAB43851), caspase-3 (1 : 1000; Bioswamp, #PAB33236), caspase-9 (1 : 1000; Bioswamp, #PAB40626), Bax (1 : 1000; Bioswamp, #PAB37588), Bcl-2 (1 : 1000; Bioswamp, #PAB30041), PI3K (1 : 1000; Bioswamp, #PAB30084), p-PI3K (1 : 1000; Bioswamp, #PAB43641-P), Akt (1 : 1000; Bioswamp, #PAB30596), p-Akt (1 : 1000; Bioswamp, #PAB43181-P), mTOR (1 : 1000; Bioswamp, #PAB30674), p-mTOR (1 : 1000; Bioswamp, #PAB43425-P), NaK-ATPase (1 : 1000; Cell Signaling Technology, #3010, Danvers, MA, USA), or GAPDH (1 : 1000; Bioswamp, #PAB36269) was added to react for 1 h with protein bands in the membranes, followed by 1 h of incubation with HRP-conjugated secondary antibody (1 : 10000; Bioswamp; #SAB43714). After visualization with chemiluminescent HRP substrate (Millipore), band intensities were analyzed by GIS Gel Image System (TANON, Shanghai, China).

### 2.6. Immunofluorescence Assay

CLIC1 and CLIC2 expression levels were examined by Immunofluorescence assay. Briefly, the cells grown in 12-well plates were washed twice with PBS, fixed with 4% paraformaldehyde for 30 min, permeabilized with 0.5% Triton X-100 (Solarbio) for 20 min, and blocked with 5% bovine serum albumin (BSA; Solarbio) at 37°C for 1 h. Afterwards, the cells were reacted with primary antibody against CLIC1 (1 : 200; Bioswamp; #PAB31716) or CLIC2 (1 : 200; Abcam; #ab175230) at 4°C overnight, followed by 1 h of incubation with Alexa Fluor 594-labeled secondary antibody (1 : 200; Bioswamp; #SAB43732) at 37°C. Then, the cells were incubated with antifade mounting medium with 4′,6-diamidino-2-phenylindole (DAPI; Solarbio) and images were taken under an inverted fluorescence microscope (Leica).

### 2.7. Measurement of Intracellular Chloride Concentration by Flow Cytometry

Intracellular chloride concentration was measured using chloride-sensitive dye N-(ethoxycarbonylmethyl)-6-methoxyquinolinium bromide (MQAE) (Beyotime, #S1082, Beijing, China) by flow cytometry according to the manufacturer's instructions. Briefly, PBS-washed cells were loaded with 5 mM MQAE at 4°C for 30 min in the dark. Then, the cells were washed 5 times with PBS and subjected to flow cytometry (ACEAbio, Santa Clara, CA, USA).

### 2.8. Evaluation of Cell Apoptosis by Flow Cytometry

Apoptosis was analyzed using PE Annexin V Apoptosis Detection Kit I (BD, #559763, San Jose, CA, USA) according to the manufacturer's instructions. Briefly, the cells were harvested by centrifugation at 400 × g and then washed once with PBS. After that, the cells were resuspended in 200 *μ*L PBS mixed with 5 *μ*L Annexin V-PE and 5 *μ*L 7-Amino-Actinomycin (7-AAD). Subsequently, the mixture was incubated in the dark (4°C, 30 min) and analyzed by flow cytometry (ACEAbio).

### 2.9. Statistical Analysis

Data were expressed as mean ± standard deviation (SD). Statistical analysis was conducted using ANOVA followed by Tukey's test. *P* < 0.05 was defined as statistically significant. All experiments were repeated independently three times.

## 3. Results

### 3.1. Construction of Recombinant Plasmids Carrying Wild-Type and Mutant SLC26A4

To investigate the effects of these mutants on the function of SLC26A4 gene and possible mechanism of these mutants in hearing loss, SLC26A4 mutants were inserted into pEGFP-N1 to generate mutant 1 (c.85G>A), mutant 2 (c.2006A>T), and mutant 3 (c.853G>A). Meanwhile, wild-type SLC26A4 was inserted into pEGFP-N1 to serve as the corresponding control. DNA sequencing analysis revealed that the G>A substitution at nucleotide 85 of SLC26A4 resulted in amino acid change at codon 29 (p.E29K) (Figure 1(a)). Additionally, the A>T transition at nucleotide 2006 and the G>A transition at nucleotide 853 resulted in amino acid substitution at codon 669 (p.D669V) (Figure 1(b)) and 285 (p.V285I) (Figure 1(c)), respectively.

### 3.2. Transient Transfection of HEK-293T Cells with Wild-Type and Mutant SLC26A4

Then, mutant 1, mutant 2, and mutant 3, as well as wild-type SLC26A4, were transiently transfected into HEK-293T cells using Lipofectamine 2000. The eukaryotic expression vector pEGFP-N1 encoded green fluorescent protein (GFP). Thus, a fluorescence microscope was used to observe GFP fluorescence in these cells. The results revealed that HEK-293T cells transfected with empty vector pEGFP-N1, wild-type SLC26A4, mutant 1, mutant 2, or mutant 3 exhibited more obvious GFP fluorescence (Figure 1(d)). In addition, after transfected plasmids 24 h and 48 h, compared with the control group, the protein levels of GFP have significant increase in vector group, wild-type group, mutant 1 group, mutant 2 group, and mutant 3 group (*P* < 0.01) (Figure 1(e)). Interestingly, compared with the vector group, the SLC26A4 mRNA expression has significant increase in wild-type group, mutant 1 group, mutant 2 group, and mutant 3 group (*P* < 0.01), but in mutant 1 group and mutant 3 group, the SLC26A4 mRNA expression was lower than wild-type group and mutant 2 group (Figure 1(f)). These results indicated that the plasmids of SLC26A4 (wild-type), SLC26A4 (E29K mutant), SLC26A4 (D669V mutant), and SLC26A4 (V285I mutant) were successfully transfected in HEK-293T cells.

### 3.3. The Effects of SLC26A4 Mutations in Cell's Pendrin and Chloride

After transfected with wild-type SLC26A4, compared with the vector group, the protein levels of membrane pendrin and cytoplasm pendrin have significant increase in wild-type group (*P* < 0.01). SLC26A4 mutations led to significant reduction in membrane pendrin, while cytoplasmic levels of pendrin significantly increased as compared to those of the wild-type group (*P* < 0.01) (Figure 2(a)). Compared with the control group, chloride concentration has significant decrease in wild-type group (*P* < 0.01) (Figure 2(b)). Compared with the wild-type group, chloride concentration has significant increase in mutant 1 group, mutant 2 group, and mutant 3 group (*P* < 0.01) (Figure 2(b)). Furthermore, we found that transfection with wild-type SLC26A4 greatly upregulated CLIC1 and CLIC2 levels compared to the vector. However, as compared to the wild-type, SLC26A4 mutants decreased both CLIC1 and CLIC2 expression (Figure 3). These results indicated that SLC26A4 mutations induce the transfer of pendrin from cell membrane to cytoplasmic, decrease chloride channel proteins, and increase chloride concentration.

### 3.4. The Effects of SLC26A4 Mutations in Cell Apoptosis and PI3K/Akt/mTOR Pathway

In wild-type group, cell apoptosis rate lower than vector group, compared with the wild-type group, cell apoptosis rate has significant increase in mutant 1 group, mutant 2 group, and mutant 3 group (*P* < 0.01) (Figure 4(a)). Meanwhile, compared with the vector group, the protein levels of caspase-3, caspase-9, and Bax were greatly downregulated, while Bcl-2 levels were upregulated in wild-type group (*P* < 0.01); compared with the wild-type group, the protein levels of caspase-3, caspase-9, and Bax were greatly upregulated, while Bcl-2 levels were downregulated in mutant 1 group, mutant 2 group, and mutant 3 group (*P* < 0.01) (Figure 4(b)). The results indicated that SLC26A4 decreases cell apoptosis, and SLC26A4 mutations induce cell apoptosis. And finally, we found that p-PI3K/PI3K, p-Akt/Akt, and p-mTOR/mTOR ratios were significantly higher in wild-type group, compared with the vector group (*P* < 0.01). However, compared with the vector group, the ratios of p-PI3K/PI3K, p-Akt/Akt, and p-mTOR/mTOR were decreased in mutant 1 group, mutant 2 group, and mutant 3 group (*P* < 0.01) (Figure 5). This means that SLC26A4 mutations can be suppressed the PI3K/Akt/mTOR pathway.

## 4. Discussion

Our previous study has reported two novel mutations (c.85G>A and c.853G>A) and one reported mutation (c.2006A>T) in SLC26A4 in children with non-syndromic hearing loss compared to normal controls (data not shown). However, whether these mutations in SLC26A4 are related to hearing loss remains unknown. In the present study, we intended to investigate the relationship between SLC26A4 mutations and hearing loss and to further clarify the possible underlying mechanism.

To investigate the possible role of these three mutations in hearing loss, SLC26A4 mutants were made by a commercial kit and then inserted into pEGFP-N1 vector. These plasmids were subjected to DNA sequencing. In this study, DNA sequencing analysis suggests that we successfully obtained recombinant plasmids carrying wild-type SLC26A4, mutant 1 (c.85G>A), mutant 2 (c.2006A>T), and mutant 3 (c.853G>A). pEGFP-N1, a eukaryotic expression vector encoding GFP, is commonly used to detect the expression of inserted genes via examination of GFP by fluorescence microscopy and Western blot [16]. After transfection of HEK-293T cells with these plasmids, we found that HEK-293T cells transfected not only with empty vector but also with wild-type SLC26A4 and mutants exhibited obvious GFP fluorescence and upregulated GFP expression compared to control cells, indicating successful transfection of these plasmids. Then, qRT-PCR was performed to verify SLC26A4 expression in HEK-293T cells. Transfection with wild-type and mutant SLC26A4 significantly upregulated SLC26A4 levels compared to the vector. These results demonstrated that wild-type SLC26A4 and all mutants were successfully transfected into HEK-293T cells and overexpressed SLC26A4 in the cells.

Pendrin, an anion exchanger that mediates the transportation of chloride, iodide, bicarbonate, and formate, is localized at the plasma membrane [17]. Generally, transmembrane proteins synthesized by ribosomes translocate from the ER to the Golgi apparatus via transport vesicles and then anchor to the plasma membrane [18, 19]. Then, membrane and cytoplasmic pendrin levels were determined. We found that transfection with wild-type SLC26A4 significantly increased pendrin levels in both plasma membrane and cytoplasm compared to vector-transfected cells. Mutations in SLC26A4 abolished the recruitment of pendrin mutants to the plasma membrane in HEK-293T cells. Similar findings are reported by previous studies [20]. In non-syndromic hearing loss patients, p.L445W and p.M147T mutations in SLC26A4,followed by cell experiments, proved that the mutation prevented pendrin from targeting to the plasma membrane [21]. This may be a crucial mechanism of Pendred syndrome [20, 22]. All the three SLC26A4 mutants may inhibit localization of Pendrin to the plasma membrane and they may be degraded via the ERAD pathway. Further studies are required to verify our hypothesis.

Pendrin, a chloride/bicarbonate exchanger with higher affinity for chloride, bicarbonate, and iodide, participates in regulation of chloride reabsorption and bicarbonate secretion [23]. To investigate whether SLC26A4 mutants affect chloride reabsorption, we examined the concentration of intracellular chloride with MQAE. The results showed that intracellular chloride concentrations were significantly elevated by wild-type SLC26A4, while reduced by SLC26A4 mutants in HEK-293T cells, which is consistent with previous study [24]. CLIC1 and CLIC2, two members of chloride intracellular channel family, are evolutionary conserved proteins and possess chloride channel activity [25, 26]. However, no study has reported the relationship between SLC26A4 mutation and CLIC proteins. Maybe CLIC1 and CLIC2 are downstream regulators of SLC26A4. In our study, CLIC1 and CLIC2 expression were examined by Immunofluorescence assay. We found that wild-type SLC26A4 increased both CLIC1 and CLIC2 expression, while mutations in SLC26A4 decreased in their levels in HEK-293T cells. These results suggest that SLC26A4 mutants may directly reduce intracellular chloride concentration or indirectly regulate this via CLIC1 and CLIC2.

Apoptosis, a form of programmed cell death that is critical for tissue homeostasis, is regulated by extrinsic and intrinsic (mitochondrial/ER) pathways [27]. It has been reported that apoptosis of cochlear hair cells is associated with hearing loss [28]. Tang et al. have revealed that highly expressed SLC26A4 is associated with inhibition of cardiomyocyte apoptosis [29]. However, whether mutations in SLC26A4 result in hearing loss through regulation of cell apoptosis remains unknown. Interestingly, apoptosis was inhibited by wild-type SLC26A4. We also found that SLC26A4 mutants significantly promoted cell apoptosis compared to the wild-type, indicating that mutations in SLC26A4 may be associated with cell apoptosis. Upon apoptotic stress, Bax and Bak are oligomerized in the mitochondrial outer membrane, resulting in cytochrome c release and subsequent activation of caspase-9/-3. Bax/Bak oligomerization during apoptosis can be suppressed by anti-apoptotic protein Bcl-2 [30]. As expected, wild-type SLC26A4 decreased caspase-3, caspase-9, and Bax levels, whereas increased Bcl-2 levels in HEK-293T cells. SLC26A4 mutants markedly increased pro-apoptotic protein levels whereas decreased anti-apoptotic protein levels. These results suggest that regulation of cell apoptosis may be an important mechanism of SLC26A4 mutants in hearing loss.

The PI3K/Akt/mTOR signaling pathway plays an important role in cell proliferation, metabolism, and metastasis [31]. Moreover, activation of the Akt/mTOR pathway contributes to cochlear hair cell regeneration [15]. However, whether SLC26A4 mutants result in hearing loss via the PI3K/Akt/mTOR pathway remains unknown. In our study, we found that wild-type SLC26A4 significantly activated, while SLC26A4 mutants inhibited the PI3K/Akt/mTOR pathway in HEK-293T cells, suggesting that this pathway may be another important mechanism of SLC26A4 mutants in hearing loss. Mounting evidences have revealed that GSK-3*β* inhibition attenuates cochlear destruction and hearing loss *in vivo* [32, 33]. Moreover, SLC26A4 can regulate GSK-3*β* expression in H9c2 cells [29]. Maybe the GSK-3*β* signaling pathway is involved in hearing loss induced by SLC26A4 mutants and this hypothesis needs to be verified.

In conclusion, wild-type SLC26A4 increased membrane and cytoplasmic pendrin, intracellular chloride concentration, and CLIC1 and CLIC2 expression. Cell apoptosis was inhibited and the PI3K/Akt/mTOR signaling pathway was activated by wild-type SLC26A4. However, SLC26A4 mutants abolished membrane targeting, reduced intracellular chloride concentration, decreased CLIC1 and CLIC2 expression, enhanced cell apoptosis, and suppressed the PI3K/Akt/mTOR signaling pathway. The present study elucidated the possible mechanism and provides novel therapeutic strategy for hearing loss due to mutations in SLC26A4.

## Figures and Tables

**Figure 1:** Sequence electropherograms and measurements of GFP and SLC26A4. (a) Mutant 1 of SLC26A4 (c.85G>A) and its corresponding wild-type sequence. (b) Mutant 2 of SLC26A4 (c.2006A>T) and its corresponding wild-type sequence. (c) Mutant 3 of SLC26A4 (c.853G>A) and its corresponding wild-type sequence. Arrows showed mutation sites in SLC26A4. (d) GFP fluorescence was observed under a fluorescence microscope after transient transfection. (e) GFP expression was determined by Western blot. GAPDH served as an internal control. (f) SLC26A4 expression was determined by qRT-PCR. GAPDH served as an internal control. ^&&^*P* <0.01 compared to the control group. ^##^*P* < 0.01 compared to the vector group.

**Figure 2:** Mutations in SLC26A4 abolish membrane targeting and decrease intracellular chloride concentration. (a) Membrane and cytoplasmic pendrin levels were measured by Western blot. NaK-ATPase and NAPDH served as internal controls for membrane and cytoplasmic proteins, respectively. (b) Intracellular chloride concentration was measured using chloride-sensitive dye MQAE.^##^*P* < 0.01 compared to the vector group. ^∗∗^*P* < 0.01 compared to the wild-type group.

**Figure 3:** Mutations in SLC26A4 downregulate CLIC1 and CLIC2 expression. The levels of CLIC1 and CLIC2 were analyzed by Immunofluorescence assay.

**Figure 4:** Mutations in SLC26A4 promote cell apoptosis. (a) Annexin V-PE/7-AAD staining assay combined with flow cytometry was performed to assess cell apoptosis. (b) The levels of caspase-3, caspase-9, Bax, and Bcl-2 were determined by Western blot. GAPDH served as an internal control. ^#^*P* < 0.05, ^##^*P* < 0.01 compared to the vector group. ^∗∗^*P* < 0.01 compared to the wild-type group.

**Figure 5:** Mutations in SLC26A4 suppress the PI3K/Akt/mTOR signaling pathway. The phosphorylated and total levels of PI3K, Akt, and mTOR were examined by Western blot. The ratios of p-PI3K/PI3K, p-Akt/Akt, and p-mTOR/mTOR were calculated. GAPDH served as an internal control. ^##^*P* < 0.01 compared to the vector group. ^∗∗^*P* < 0.01 compared to the wild-type group.

## Data Availability

The data used to support the findings of this study are available from the corresponding author upon request.
